# Potential Progression Mechanism and Key Genes in Early Stage of mTBI

**DOI:** 10.1155/2022/3151090

**Published:** 2022-08-03

**Authors:** Hu Zhou, Xue Han, Hui-xia Zhou, Zhen-zhen Cao, Li Yang, Jian-yun Yu

**Affiliations:** ^1^Department of Forensic Medicine, Kunming Medical University, Kunming 650500, Yunnan, China; ^2^Department of Neurosurgery, The First People's Hospital of Yunnan Province, Kunming 650032, Yunnan, China; ^3^Department of Tissue Embryology and Anatomy, Kunming Medical University, Kunming 650500, Yunnan, China

## Abstract

Chronic traumatic encephalopathy (CTE) is a neurodegenerative disease caused by repetitive mild traumatic brain injury (rmTBI), and the lack of sensitive diagnostic and prognostic biomarkers for rmTBI leads to long-term sequelae after injury. The purpose of this study is to identify key genes of rmTBI and find the potential progression mechanism in early stage of mTBI. We downloaded the gene expression profiles of GSE2871 from Gene Expression Omnibus (GEO) datasets. Differentially expressed genes (DEGs) were screened from the cerebral cortex of rats 24 hours after smTBI, and these DEGs were then subjected to GO enrichment analysis, KEGG pathway analysis, PPI analysis, and hub analysis. Key genes were identified as the most significantly expressed genes and had a higher degree of connectivity from hub genes. By using homemade metal pendulum impact equipment and a multiple regression discriminant equation to assess the severity of rats after injury, smTBI and rmTBI rat models were established in batches, and q-PCR analyses were performed to verify the key genes. The main KEGG pathways were cytokine-cytokine receptor interaction and neuroactive ligand-receptor interaction. SPP1 and C3 were the most significant DEGs, and their connectivity degree was the highest 24 hours after smTBI (logFC > 4; connectivity degree ＞15). The q-PCR analyses were performed 24 hours and 14 days after mTBI. The results showed that SPP1 and C3 were significantly upregulated in smTBI and in rmTBI at 24 hours after injury compared with their levels in sham-injured rats, and the phenomenon persisted 14 days after injury. Notably, 14 days after injury, both of these genes were significantly upregulated in the rmTBI group compared with the smTBI. These pathways and genes identified could help understanding the development in mTBI.

## 1. Introduction

Traumatic brain injury (TBI) is a global public health problem, and its incidence is increasing [1]. TBI is one of the leading causes of death and dysfunctions. Patients also experience associated cognitive, emotional, physical, and sensory disabilities, which often result in quality-of-life reductions and job losses. [2] Mild TBI (mTBI) is the leading cause of death and disabilities in the United States and worldwide, with approximately 42 million cases annually [3]. Patients may present a complex array of symptoms, including cognitive disturbance, physical fatigue, decreased sleep quality [4], and depression or migraine [5]. Further insights into the underlying biological injury should be obtained, and the identification of key genes is essential for finding biomarkers and therapeutic targets for the mTBI. Studies have shown that IL-1*α*, IL-8, and IL-6 [6] and the glycolytic enzyme neuron-specific enolase (NSE) are biomarkers for the mTBI [7] and are involved in various biological processes, including the inflammatory response and hormone regulation. Secondary brain injury after TBI is very complex, and more valuable biomarkers need to be identified. Furthermore, the study of biomarkers for repetitive mTBI (rmTBI) is essential for the understanding and treatment of the chronic traumatic encephalopathy. Unfortunately, the genes that show significantly differential expression after the rmTBI have not been studied, and studying the gene profile of single mTBI (smTBI) is an alternative approach for exploring the key genes of rmTBI.

In this paper, we identified differentially expressed genes (DEGs) by comparing mTBI with sham-injured rats to determine the key biological processes and pathways associated with these DEGs. We constructed a protein-protein interaction network and screened the hub genes from these DEGs. The genes with the highest fold-change were selected and validated by a q-PCR analysis of the frontal cortex of a rat model of mild brain injury. In this study, the accumulative effect was explored by comparing the expression of these genes in rats with rmTBI with that in rats with smTBI, and the expression of these genes at different time points was also studied to identify biomarkers of rmTBI. This information might provide further insights into the mechanism underlying the progression of mTBI and might identify potential therapeutic targets for mTBI. A total of 123 upregulated genes and 88 downregulated genes were identified. The biological processes of DEGs were mainly involved in the negative regulation of immune system processes and regulation of immune effector processes. The following are the major contributions of the research conducted in this paper: (1) key genes of rmTBI are identified, and the potential progression mechanism in the early stage of mTBI is found; (2) the accumulative effect was explored by comparing the expression of these genes in rats with rmTBI with that in rats with smTBI; and (3) the expression of these genes at different time points was also studied to identify biomarkers of rmTBI.

The rest of the paper is organized as follows. In Section 2, we offer an overview of the materials and methods.  Section 3 is about the datasets and evaluation metrics. Moreover, experimental details are also presented. In Section 4, results are discussed along with the related work. Finally, Section 5 concludes this paper and offers several directions for further research and investigation.

## 2. Materials and Methods

### 2.1. Data Source

The GSE2871 was downloaded from the Gene Expression Omnibus (GEO) database available online (https://www.ncbi.nlm.nih.gov/, downloaded on 06/03/2019) [8]. This dataset comprises 47 samples, including two samples from the ipsilateral cortex of sham-injured rats and two samples from the ipsilateral cortex of rats with mTBI. We then compared the mTBI samples with the sham samples to identify DEGs.

### 2.2. Data Processing

First, the “impute” package in R [9] was used to supplement the missing values in the mRNA expression data, and the raw data were preprocessed identically using the “limma” package in R [10] to identify the DEGs between the mTBI and sham groups based on the criteria |logFC| ≥ 1.0 and *p* value <0.05. Volcano plots of all the genes and heat maps are presented.

### 2.3. Gene Ontology (GO) Functional Annotation and Kyoto Encyclopedia of Genes and Genomes (KEGG) Pathway Analysis of DEGs

AGO enrichment analysis was performed to analyze the biological process (BP), molecular function (MF), and cellular component (CC) of DEGs. The pathways associated with the DEGs were identified by KEGG pathway analysis. These analyses could provide a better understanding of the metabolic pathways of TBI. GO functional annotation and KEGG pathway analysis of the DEGs, identified in this study, were performed using the “cluster Profiler” package in the R statistical language [11]. KEGG pathway analysis of the DEGs identified in our study was performed using the “pathview” package in the R [12]. The genes meeting the criteria adjusted *p* < 0.05 and gene counts ≥10 were significantly enriched.

### 2.4. Protein-Protein Interaction Network (PPI) and Hub Genes

The Search Tool for the Retrieval of Interacting Genes (STRING) database (available online at https://string-db.org/, downloaded on 06/03/2019) was used to obtain information for establishing a protein-protein interaction network (PPI) [13]. The potential PPI relationships were obtained by searching the previously identified DEGs in the STRING database. Subsequently, we used Cytoscape software (Cytoscape 3.7.1) to construct the PPI network [14]. Nodes with higher connectivity are often critical for maintaining the stability of the network. CytoHubba, a plugin in Cytoscape software, was used to calculate the degree of each protein node [15]. In our study, the genes with the highest degree of connectivity were identified as hub genes.

### 2.5. Establishment of an Animal Model of mTBI

A total of 272-month-old male specific-pathogen-free Sprague-Dawley rats (270–300 g, purchased from the SlacJingda Experimental Animals Company [Changsha, Hunan Province, China; license No. SCXK (Xiang) 2016-0002] were randomly divided into six experimental groups (four rats per group): (i) 24-hour control sham-injured group, (ii) 24-hour post-smTBI group, (iii) 24-hour post-rmTBI group (three repeated injuries), (iv) 14-day control sham-injured group, (v) 14-day post-smTBI group, and (vi) 14-day post-rmTBI group (three repeated injuries). The mTBI rat model were established using a custom-designed device consisting of a metallic pendulum striker as described previously [16]. Each rat was placed in a stereotactic frame, and its occiput skull was impacted with a metal pendulum (1,450 grams). The rats belonging to the smTBI groups were impacted only once, and the rats belonging to the repeat mTBI groups were impacted once per day for three consecutive days. The rats in the sham injury group were exposed to the pre- and poststrike environments but were not harmed by the impact. The rats were sacrificed after 24 hours and 14 days, and the whole brain tissue was collected. Prefrontal cortex tissues were then dissected, rapidly frozen in liquid nitrogen, and stored at −80°C for PCR assay. All animal care and experimentation procedures were performed in strict accordance with the guidelines established by the National Institutes of Health, and ethical approval for the experiments was obtained from the Education Commission of Kunming Medical University.

### 2.6. Real-Time Quantitative PCR Verification

Total RNA from the prefrontal cortex tissue samples was extracted using TRIzol reagent (Invitrogen, Carlsbad, CA, USA). The concentration and purity of the total RNA were determined using spectrophotometer, and the A260/A280 values were between 1.8 and 2.0. Based on the instructions provided with the RevertAid Fist Strand cDNA Synthesis Kit (Thermo, K1622), primer sequences were synthesized, and reverse transcription was performed to generate cDNA. According to the real-time fluorescence quantitative PCR kit, a 10 *μ*L reaction system was subjected to the following reaction conditions: 10 min at 95°C, 40 cycles of 10 s at 95°C, 20 s at 60°C, and 30 s at 72°C, and cooling to 65°C. The relative mRNA expression was calculated automatically with the RT-PCR instrument.  Table 1 shows the primer sequences used for PCR amplification.

### 2.7. Statistical Analysis

GraphPad Prism 8.2 (GraphPad Prism Software, Inc., San Diego, CA, USA) was used for the statistical analyses of previously obtained experimental data. The statistical results are presented as the means ± standard deviations (SDs). Note that the symbol denotes the standard deviations (dispersion or variations). A *t* test was used to evaluate the mRNA expression levels of key genes in different tissues, and *p* < 0.05 was considered to indicate a statistically significant difference.

## 3. Results

### 3.1. Identification of DEGs

The GSE2871 dataset was processed using the “impute” and “limma” packages in the R. According to the criteria |logFC| > 1.0 and *p* < 0.05, 123 upregulated genes and 88 downregulated genes (211 in total) were identified in the comparison of the 24-hour post-smTBI group with the sham-injured mTBI group. All 5944 genes were plotted in Figure 1(a), where the red color indicates upregulated genes, the green color represents downregulated genes, and the rest of the genes are shown in black. The top 20 DEGs are presented in the heatmap, and these genes were clustered between the sham and mTBI groups, as shown in Figure 1(b).

### 3.2. Gene Ontology (GO) Enrichment Analysis and Kyoto Encyclopedia of Genes and Genomes (KEGG) Pathway Analysis of DEGs

The results of the GO function annotation analysis and KEGG pathway enrichment analysis of DEGs identified in the ipsilateral cortex are shown in Table 2 and Figures 2(a) and 2(b). The criteria used in the analysis were adjusted *p* < 0.05 and gene count ≥10. The cellular components (CC) that were significantly enriched were the external side of the plasma membrane (adjusted *p*=0.001830905, gene count = 14), the apical part of the cell (adjusted *p*=0.046821474, gene count = 11), and the apical plasma membrane (adjusted *p*=0.039668583, gene count = 11). The analysis of molecular functions (MFs) revealed that the DEGs were enriched in receptor ligand activity (adjusted *p*=1.05*E* − 06, gene count = 20), receptor regulator activity (adjusted *p*=1.93*E* − 06, gene count = 20), cytokine activity (adjusted *p*=9.44*E* − 06, gene count = 12), and cytokine receptor binding (adjusted *p*=0.004590706, gene count = 11). The biological processes (BP) of the DEGs were mainly enriched in negative regulation of the immune system process (adjusted *p*=0.000130695, gene count = 18), regulation of immune effector process (adjusted *p*=0.000182696, gene count = 16), wound healing (adjusted *p*=0.000495285, gene count = 16), response to corticosteroid (adjusted *p*=0.000122132, gene count = 15), and response to lipopolysaccharide (adjusted *p*=0.002612511, gene count = 15). The KEGG pathway analysis of the DEGs revealed particular enrichment in the cytokine-cytokine receptor interaction (adjusted *p*=0.01018118, gene count = 12), neuroactive ligand-receptor interaction (adjusted *p*=0.032342367, gene count = 12), and Epstein-Barr virus infection (adjusted *p*=0.032342367, gene count = 12).

### 3.3. PPI Network Construction and Hub Gene Identification

Protein interaction information for the DEGs identified from the cortex of rats with mTBI was predicted using STRING tools. The information was analyzed using Cytoscape software from the STRING. A total of 102 nodes and 303 edges were included in the PPI network, as presented in Figure 3. The hub genes were identified based on a connectivity degree greater than 15 in the PPI network (Table 3). The results showed that Il10 had the highest connectivity degree (degree = 25), followed by Mmp9 (degree = 22), Ccl2 (degree = 20), Spp1 (degree = 19), Timp1 (degree = 18), C3 (degree = 17), Cxcl10 (degree = 16), and Anxa1 (degree = 15). All of these hub genes were upregulated in mTBI.

### 3.4. Q-PCR Validation of the Hub Genes

SPP1 and C3 were identified as the most significantly expressed genes and had a higher degree of connectivity in the smTBI, as determined in a previous bioinformatics analysis (Table 3). To verify whether SPP1 and C3 are upregulated in the mTBI, the rats in the rmTBI group were given three strikes and observed 24 hours and 14 days after injury. At 24 hours after injury, the SPP1 and C3 expression levels were increased in both the smTBI and rmTBI groups compared with the sham-injured group, and the SPP1 and C3 expression levels showed no significant difference between the smTBI and rmTBI groups. At 14 days after injury, SPP1 and C3 expression level were increased in both the smTBI and rmTBI groups compared with the sham-injured group. In addition, the expression of SPP1 and C3 was significantly increased in the rmTBI group compared with the smTBI group. The results are shown in Figures 4 and 5.

## 4. Discussion

The mTBI is common among soldiers and athletes, and the sequelae affect their life and work. Moreover, CTE is associated with high mortality and disability rates, which makes its treatment a difficult problem in the clinic. Early intervention is crucial, and new biomarkers and therapeutic targets for the mTBI need to be identified. In this study, we comprehensively analyzed the DEGs 24 hours after smTBI. The DEGs in mTBI are mainly concentrated on the external side of the plasma membrane, the apical part of the cell, and the apical plasma membrane and are involved in a variety of biological processes, such as immune regulation, inflammatory response, regeneration, proliferation, and hormone secretion. We identified eight hub genes that might play an important role in the progression of mTBI: (1) Il10, (2) Mmp9, (3) Ccl2, (4) SPP1, (5) Timp1, (6) C3, (7) Cxcl10, and (8) Anxa1. Notably, SPP1 and C3 were most significantly upregulated, and this result was verified in vivo. Moreover, SPP1 and C3 remained significantly upregulated in the rmTBI, and the upregulation persisted 14 days after the injury. Moreover, at 14 days after injury, these two genes exerted a significant cumulative effect on rmTBI compared with their effect on the smTBI.

Secreted phosphoprotein 1 (SPP1), which is known as osteopontin, is expressed in large pyramidal neurons in the primary motor cortex of certain primate species. When injury occurs, SPP1 is expressed in response to injury and inflammatory signals, binds to receptors to promote cell chemotaxis, adhesion, and migration and participates in inflammatory and immune processes [17–19]. SPP1 expression is involved in tissue homeostasis, wound healing, immune regulation, stress response, and other injury-induced immune physiological processes, and this multifunctional protein is related to a variety of pathophysiological processes. Studies have also found that SPP1 might support nerve burst buds to promote central nervous system trauma recovery [19, 20]. Besides, previous studies have shown that SPP1 is related to the cognitive function and that SPP1 is significantly expressed in early cognitive dysfunction in Alzheimer's disease [21].

The upregulation of SPP1 can not only increase the phagocytosis of amyloid *β*-protein (A*β*) by promoting macrophage infiltration but also promote the elevation of the anti-inflammatory factors iNO, IL-10, and A*β*-degrading enzyme MMP-9 to play a neuroprotective role [22]. However, some studies have obtained the opposite findings, which suggests that SPP1 increases the levels of inflammatory markers, including IL13R1, CXCR3, and CD40L, and that local SPP1 expression combined with surrounding inflammatory stimuli might be associated with the development of inflammation in the brain and the induction of cell death [23]. Thus, further large-scale studies are needed to elucidate the role of SPP1 in neurodegenerative diseases. Tang et al. found that SPP1 was upregulated four hours after TBI. This study showed that SPP1 not only was significantly expressed at the early stages of both smTBI and rmTBI but was still significantly expressed 14 days after smTBI and rmTBI; therefore, SPP1 might be an important factor associated with the cognitive dysfunction in CTE.

Complement component 3 (C3) is a protein-coding gene, and C3 plays a central role in the activation of the complement system [24]. In particular, its activation is required for both classical and alternative complement activation pathways. The complement system is a biochemical pathway involved in both innate and adaptive immune responses and has four main functions: lysis of microorganisms, promotion of phagocytosis, triggering inflammation, and immune clearance [25, 26]. The activation of C3 can trigger a continuous degradation mechanism to activate microglia and astrocytes, reduce the density of dendritic cells and synapses, and inhibit the migration of neuroblast cells, which leads to neuron loss after several weeks of TBI [27, 28]. The upregulation of C3 can promote the progression of the neurodegenerative diseases, and previous studies have shown that C3 in turn interacts with the C3aR neurons and microglia to mediate *β*-amyloid pathology and neuroinflammation in AD mouse models. Therefore, these can further impair the cognitive function and reduce A*β* phagocytosis [29].

The synergism of C3 and APOE 4 can potentially increase amyloid deposition and Tau hyperphosphorylation in the cerebrospinal fluid of patients with Alzheimer's disease [30]. The activation of complement C3 in the human AD brain is necessary for amyloidosis and neurodegeneration caused by tau pathology. Moreover, the blocking the functions of C3 might exert protective effects in AD and neurodegenerative diseases [31–33]. In this study, C3 was significantly expressed in both the smTBI and rmTBI groups. Notably, C3 exerts an obvious accumulation effect after 14 days of the rmTBI compared with the smTBI. C3-mediated chronic inflammation might be an important mechanism for the development of repetitive mild brain injury into CTE, and the identification of the C3 gene might provide new ideas for the treatment of CTE. This study showed that mTBI induced the upregulation of SPP1 and C3, and these genes were significantly upregulated in the rmTBI to induce neurodegenerative degeneration and eventually the development of the CTE [15, 16].

## 5. Conclusions and Future Work

In this paper, we identified SPP1 and C3 as hub genes of mTBI. These genes are involved in secondary brain injury after mTBI and might be candidate biomarkers of and potential therapeutic targets in mTBI. This study showed that mTBI induced the upregulation of SPP1 and C3, and these genes were significantly upregulated in rmTBI to induce neurodegenerative degeneration and eventually the development of CTE. These pathways and genes identified could help to understand the mechanism of development in mTBI. Spp1 and C3 might be biomarkers for smTBI and rmTBI and might be turn into potential therapeutic targets for mTBI. Further studies on mTBI are needed. In particular, the mechanisms through which these genes contribute to dysfunction in CTE need to be further elucidated. We believe further large-scale studies are still needed to elucidate the role of SPP1 in neurodegenerative diseases. The limitation of this study is that though multiple therapeutic targets were identified, drug analysis was not performed, and further research on drug analysis will be conducted in the future.

## Figures and Tables

**Figure 1:** (a) Volcano plot of 5944 genes. The red dots represent upregulated genes with a fold change ≥1.0, the green dots represent downregulated genes with a fold change ≤−1.0, and the black dots represent the rest of the genes that showed no significant change in expression. (b) Heatmap of the top 20 differentially expressed genes. The red color represents upregulation, and the green color indicates downregulation. Figures 1(a) and 1(b) show that SPP1 and C3 were the most significantly differentially expressed genes in smTBI and were upregulated.

**Figure 2:** (a) Gene ontology (GO) enrichment analysis of differentially expressed genes (DEGs). (b) Kyoto encyclopedia of genes and genomes (KEGG) pathway analysis of DEGs. The *Y*-axis represents gene functions, and the *X*-axis represents gene ratios. Each bar represents a different enrichment function, and the significance threshold was set to adjusted *p* < 0.05.

**Figure 3:** PPI network of the DEGs in smTBI. The red nodes indicate upregulated genes, the green nodes indicate downregulated genes, and the node size is correlated with the degree of connectivity of the gene.

**Figure 4:** Comparison of SPP1 mRNA levels in the frontal cortex of rats. (a)–(c) Identification of the SPP1 gene identified 24 hours post mTBI. (a) Validation of the changes in the SPP1 mRNA expression level between the sham and smTBI groups. (b) Validation of the changes in the SPP1 mRNA expression level between the sham and rmTBI groups. (c) Validation of the changes in the SPP1 mRNA expression level between the smTBI and rmTBI groups. (d)–(f) Identification of the SPP1 gene 14 days after mTBI. (d) Validation of the changes in the SPP1 mRNA expression level between the sham and smTBI groups. (e) Validation of the changes in the SPP1 mRNA expression level between the sham and rmTBI groups. (f) Validation of the changes in the SPP1 mRNA expression level between the smTBI and rmTBI groups. The data are presented as the means ± SDs, and *p* < 0.05 was considered to indicate significance. smTBI: single mild traumatic brain injury; rmTBI: repetitive mild traumatic brain injury.

**Figure 5:** Comparison of C3 mRNA levels in the frontal cortex of rats. (a)–(c) Identification of the C3 gene 24 hours after mTBI. (a) Validation of the changes in the C3 mRNA expression level between the sham and smTBI groups. (b) Validation of the changes in the C3 mRNA expression level between the sham and rmTBI groups. (c) Validation of the changes in the C3 mRNA expression level between the smTBI and rmTBI groups. (d)–(f) Identification of the C3 gene 14 days after mTBI. (d) Validation of the changes in the C3 mRNA expression level between the sham and smTBI groups. (e) Validation of the changes in the mRNA expression level between the sham and rmTBI groups. (f) Validation of the changes in the C3 mRNA expression level between the smTBI and rmTBI groups. The data are presented as the means ± SDs, and *p* < 0.05 was considered to indicate significance. smTBI: single mild traumatic brain injury; rmTBI: repetitive mild traumatic brain injury.

**Table 1:** Primer sequences for polymerase chain reaction amplification.

Gene	Sequence
SPP1	Forward: 5′-GGT TTG CTT TTG CCT GTT CG-3′
	Reverse:5′-GCT CTC TGC ATG GTC TCC GT-3′
C3	Forward: 5′-AAG CAT CAA CAC ACC CAA CA-3′
	Reverse:5′-CTT GAG CTC CAT TCG TGA CA-3′
GAPDH	Forward: 5′-GCA AGA GAG AGG GCC CTC AG-3′
	Reverse:5′-TGT GAG GGA GAT GCT CAG TG-3′

**Table 2:** Gene ontology (GO) and KEGG pathway enrichment analysis of differentially expressed genes (DEGs) with adjusted *p* < 0.05 and gene counts ≥10.

Category	ID	Term	Adjusted *p*	Count
Biological process	GO: 0002683	Negative regulation of immune system process	0.000130695	18
Biological process	GO: 0002697	Regulation of immune effector process	0.000182696	16
Biological process	GO: 0042060	Wound healing	0.000495285	16
Biological process	GO: 0031960	Response to corticosteroid	0.000122132	15
Biological process	GO: 0032496	Response to lipopolysaccharide	0.002612511	15
Biological process	GO: 0008202	Steroid metabolic process	0.000130695	14
Biological process	GO: 0051384	Response to glucocorticoid	0.000130695	14
Biological process	GO: 0019216	Regulation of lipid metabolic process	0.000725406	14
Biological process	GO: 0002443	Leukocyte mediated immunity	0.001029513	14
Biological process	GO: 0001819	Positive regulation of cytokine production	0.003130079	14
Biological process	GO: 0070661	Leukocyte proliferation	0.000819502	13
Biological process	GO: 0007584	Response to nutrient	0.002465097	13
Biological process	GO: 0001525	Angiogenesis	0.00904787	13
Biological process	GO: 1903532	Positive regulation of secretion by cell	0.00914943	13
Biological process	GO: 0050777	Negative regulation of immune response	4.29*E* − 05	12
Biological process	GO: 0051048	Negative regulation of secretion	0.000819502	12
Biological process	GO: 0031099	Regeneration	0.002267839	12
Biological process	GO: 0050727	Regulation of inflammatory response	0.003740474	12
Biological process	GO: 0002250	Adaptive immune response	0.004711657	12
Biological process	GO: 0022407	Regulation of cell-cell adhesion	0.006702972	12
Biological process	GO: 0002698	Negative regulation of immune effector process	4.72*E* − 05	11
Cellular component	GO: 0009897	External side of plasma membrane	0.001830905	14
Cellular component	GO: 0045177	Apical part of the cell	0.046821474	11
Cellular component	GO: 0016324	Apical plasma membrane	0.039668583	10
Molecular function	GO: 0048018	Receptor ligand activity	1.05*E* − 06	20
Molecular function	GO: 0030545	Receptor regulator activity	1.93*E* − 06	20
Molecular function	GO: 0005125	Cytokine activity	9.44*E* − 06	12
Molecular function	GO: 0005126	Cytokine receptor binding	0.004590706	11
KEGG pathway	rno04060	Cytokine-cytokine receptor interaction	0.01018118	12
KEGG pathway	rno04080	Neuroactive ligand-receptor interaction	0.032342367	12
KEGG pathway	rno05169	Epstein-barr virus infection	0.032342367	10

**Table 3:** Eight hub genes with connectivity degree ≥15 identified from the differentially expressed genes (DEGs) in mTBI.

Gene symbol	Gene description	Degree	logFC	*p*-value
Il10	Interleukin 10	25	2.051802	0.012652
Mmp9	Matrix metallopeptidase 9	22	1.044537	0.011024
Ccl2	C-C motif chemokine ligand 2	20	1.812989	0.01822
Spp1	Secreted phosphoprotein 1	19	4.354135	4.77E-05
Timp1	TIMP metallopeptidase inhibitor 1	18	1.513157	0.031929
C3	Complement component 3	17	4.17003	0.001008
Cxcl10	C-X-C motif chemokine ligand 10	16	1.085489	0.014918
Anxa1	Annexin A1	15	1.355688	0.011361

## Data Availability

All data generated or analyzed during this study are included within thepublished article.
